# Prepayment Model of Supply Chain Financing Based on Internet of Things and Machine Learning Algorithm

**DOI:** 10.1155/2022/9320692

**Published:** 2022-08-21

**Authors:** Zhaohui Duan

**Affiliations:** Hebei Chemical & Pharmaceutical College, Shijiazhuang, Hebei 050030, China

## Abstract

Nowadays, the relationship between all kinds of things is constantly strengthened, and the regional restrictions on things are also constantly weakened, especially in the aspect of trade. In the past, people could only buy some basic goods in a relatively small area if they wanted to buy them in a relatively small area, but now the situation is very different. People's dependence on traders is gradually decreasing; that is to say, the traditional advantages of traders are gradually losing. Particularly, in today's fierce competition, survival of the fittest, and limited profits, the entire trade industry is facing a lot of impacts, not to mention the survival of traders relying on this industry. Therefore, traders must think of a new way to adapt to the characteristics of the new era, to continue to make profits and maintain their own survival. In fact, for the whole industry, this is also the most urgent problem to be solved. This study mainly explores the above problems and puts forward some feasible methods to solve the problems, hoping to cause some thinking of the industry personnel, so that they can modify and adjust their working mode. In addition, it should be emphasized that the mode of using Internet of things and machine learning to achieve the purpose of innovation is of great practical significance.

## 1. Introduction

Due to the development of Internet technology, online shopping has become a new shopping trend [1]. In contrast, the traditional form of shopping has been impacted, and the business model has to adapt to the times. To survive in all kinds of fierce competition, upstream suppliers take many measures, such as purchasing other suppliers to increase their core competitiveness, so as to occupy more resources and markets and earn more profits [2]. However, for downstream enterprises and end users, their methods are slightly different. Generally speaking, they will use various interpersonal relationships to directly trade with upstream suppliers through various channels, so as to reduce costs and increase profits as much as possible [3]. With the development and progress of society, the trade industry has also undergone great changes, one of which is that its entry threshold is lower, but the competition has become more intense. Generally speaking, that is to say, nowadays more and more people can do business, but at the same time, due to the increasing sales channels of various commodities, the competition in sales is also in increasingly fierce [4]. For trading companies, they are in the middle of the whole sales chain and are often restricted by many factors, such as small price adjustment range, small external demand, and fierce competition in all aspects, and now, the advantages of traders in the past are also shrinking, eventually leading to the continuous reduction in their profits, facing a grim situation [5]. However, these thorny problems are not insurmountable. For example, some domestic commercial banks put forward the supply chain financial service scheme, which can perfectly deal with the problem of difficult access to funds in many small- and medium-sized enterprises [6]. Based on this perspective, this study analyzes the advantages and disadvantages of financing services provided by banks and possible problems and risks from the perspective of obtaining funds using Internet of things and machine learning, to explore the cost-benefit situation of supply chain under the mode of prepayment financing and the financing decision-making scheme of banks [7].

## 2. Related Work

The literature mainly discusses multinational companies, based on these enterprises to discuss the financing problem between them and suppliers [8]. Considering that compared with these multinational companies, generally speaking, suppliers are smaller in scale and weaker in strength. Therefore, in reality, they generally cannot obtain the financing services provided by banks [9]. Without sufficient funds, these suppliers will not be able to reasonably adjust their internal operation and thus cannot reduce the production cost, which will affect to a certain extent. It affects the production cost of multinational companies and other enterprises. The first analysis in the literature is the development of supply chain financing [10]. Through the research, we found that there are two shortcomings: first, it does not fully consider the logistics and capital flow. After further practical research, we find that most of the existing supply chain financing focuses on logistics, but ignores it. The importance of capital flow ultimately leads to the reduction in the role of supply chain financing; second, the cost remains high due to the failure to form a strict and scientific financial system between the buyer and the seller. To sum up, the literature suggests that we should use the existing science and technology to establish a sound financial system and reasonably adjust the industry's attention to capital flow issues, so as to improve the supply chain financing [11]. The literature established a suitable model to analyze how to optimize the existing supply chain and finally reached the following conclusion: only by sharing information we can solve the problem of high cost and play the largest role of supply chain financing [12]. The literature also establishes a model according to the actual situation to explore the intuitive understanding of the supply chain capital flow [13]. However, in reality, it is much more complicated than the model, and it is often impossible to determine which account this income corresponds to. In other words, we cannot find the exact capital flow between income and expenditure. The reference focuses on the relationship between suppliers and sellers in the supply chain [14]. After the relevant research found that if they want to reduce their costs, they must work together to solve the problem, so as to achieve mutual benefit and win-win situation. The literature also uses the method of establishing a model for analysis and research and finally puts forward the following conclusions: if SMEs want to obtain profits, they must find the core enterprises that can be trusted and establish a relatively long and stable cooperation mode with them [15]. The literature suggests to reduce the related risk by shortening the cash conversion cycle as much as possible [16]. The literature once again emphasizes the use of electronic information technology in the operation of supply chain [17].

## 3. Related Technology and Theoretical Basis

### 3.1. Main Operation Modes of Supply Chain Financing

As far as the actual situation is concerned, the operation of domestic supply chain financing is mainly in the charge of banks, which provide liquidity financing to relevant enterprises under the condition of ensuring their repayment ability. Moreover, considering the different repayment ability of different enterprises, the financing schemes provided by banks are also different. This study analyzes the supply chain financing mode of the more authoritative banks nowadays. The most widely used are the following three modes: accounts receivable operation mode, confirmed warehouse operation mode, and financing warehouse operation mode.

#### 3.1.1. There Are Two Financing Schemes for Accounts Receivable Financing, Which Have Different Operation Modes

The first scheme is the pledge of accounts receivable. In this way, the enterprise takes its own sales revenue as the first source of funds to repay the bank, and the bank mainly judges its credit when considering whether to provide funds to the enterprise. The second scheme is the transfer of accounts receivable. Its actual operation is completely different from the previous one. This scheme has specific debtors, and the enterprise needs to open a special account in the bank to repay the borrowed funds, which can be directly remitted into this special account. Of course, it is not to say that the two schemes have nothing in common. In fact, both of them require banks to review the whole supply chain as the credit subject, which reduces many risks and greatly ensures the safety of bank financing.  Figure 1 shows the business process of pledge of accounts receivable as an example.

People transfer accounts receivable, that is, factoring business. After the seller and the factor sign the accounts receivable transfer agreement, it has the qualification to transfer it not yet due to qualified accounts receivable to the factor. Generally speaking, factoring agents, that is, banks, can not only provide financing but also serve enterprises in many other aspects, such as account management. Factoring is generally divided into international factoring and domestic factoring according to the geographical scope involved.

#### 3.1.2. Operation Mode of Confirmed Warehouse

As the name implies, the buyer is in the upper position of the whole supply chain. When it prepays the following enterprises, if the funds are paid through bank financing, then this is called confirmed warehouse operation mode, that is, prepayment operation mode. The specific business process is shown in Figure 2.

#### 3.1.3. Operation Mode of Financing Warehouse

In theory, the financing warehouse is divided into two types according to the practical operation mode: the first is called the credit guarantee operation mode. In this mode, the commercial banks regard the logistics and warehousing enterprises as credit enterprises, then evaluate their repayment ability by considering the characteristics and capabilities of various aspects of the enterprises, and then provide them with appropriate supply chain financing services. It can screen out the enterprises that it trusts and has a long-term cooperative relationship to provide relevant guarantee for it, so as to increase its credit strength; the second is called pledge guarantee operation mode, which is different from the previous one. Banks regard enterprises with long-term cooperative relationship with logistics enterprises as credit enterprises and then provide appropriate credit for cooperative enterprises after evaluation as for the enterprise's repayment fund, and it depends on the return of selling inventory goods.

### 3.2. Application Principle of Internet of Things Technology in Prepayment Mode of Supply Chain Finance

With the development of science and technology, intelligent manufacturing has become a common phenomenon. More and more enterprises begin to put intelligent equipment into production practice. Among the intelligent equipment, visual identification technology is the most widely used intelligent equipment. Through the application of visual identification technology, the whole process of production monitoring and automatic collection of production data can be realized. In addition, the reduction in the cost of science and technology also makes the application of intelligent equipment more and more widely. On the one hand, the application of intelligent equipment can reduce human and material resources, and on the other hand, it can improve the efficiency and accuracy of enterprise management, which is conducive to the development of enterprises. In the past, enterprise data collection needs a lot of manpower and the efficiency is slow, but with the application of intelligent technology, data collection becomes more and more simple. The rapid data collection and communication can be realized through the Internet, which not only ensures the efficiency of data collection but also improves the accuracy and real time of data. Now, most enterprises use intelligent devices to manage enterprise data. The use of intelligent devices enables enterprises to continuously obtain the latest data, which is conducive to the development of effective risk aversion. The functions and principles of risk aversion of intelligent devices are shown in Table 1.

### 3.3. Intelligent Analysis Method of Supply Chain Based on Machine Learning

An enterprise is a complex system, and changes in each small part will affect the status of the entire enterprise. Therefore, it is necessary to grasp the implementation of each part of the enterprise supply chain. This requires strengthening the supply chain testing during the production process. The testing methods include enterprise surveys and questionnaire surveys. This testing method can investigate the problems that occur in the actual supply chain and summarize and sort these problems to find A solution. Generally speaking, the factors that affect the supply chain during the investigation process are often also problematic factors. The problems that arise in practice can be combined with theoretical knowledge to determine the factors affecting the supply chain to form a correlation between the supply chain and the factors. Starting from the idea of axiomatic design, this study establishes the mapping relationship between the index domain *K*—factor domain *F*—problem domain *Q*, as shown in Figure 3. In fact, the information collected in this study is not enough to establish the effect standard of the supply chain. Therefore, this paper only studies the mapping relationship between supply chain influencing factors.

To determine the main factors affecting the supply chain, we should first determine the performance evaluation criteria of the supply chain, quantitatively analyze the strategic organization of the supply chain, and use the supply chain data measurement method to form a large number of sample data related to the supply chain. The above work is for supply. Data mining of key factors of the chain provides conditions. In summary, the technical route of the intelligent analysis method of supply chain performance proposed in this study is shown in Figure 4.

It can be seen from the figure that the research method proposed in this study includes the following three key technologies, the logical sequence of which is consistent with machine learning and knowledge acquisition.

## 4. Model Construction and Analysis of Supply Chain Financing Prepayment Model

### 4.1. Model Construction of Prepayment Financing Model

Among the financial models of the supply chain, prepayment is the most typical model. The entire economic flow process of the supply chain can be divided into two parts, upstream and downstream. The core of the upstream is the supplier, and the core of the downstream is the distributor. Most of the distributors in this part are small- and medium-sized enterprises. Compared with the suppliers, downstream companies are at a disadvantage in the entire supply chain. When small- and medium-sized enterprises seek financing services, they also need to contact banks through upstream enterprises, which further strengthen the disadvantaged position of SMEs. This article discusses a simple supply chain single-cycle model composed of banks, suppliers, and distributors. Now, the following assumptions are made about the model, and the relevant variables of the prepayment financing model are defined.

After entering the marketing step, the distributor first needs to speculate on the market demand in order to place an order with the supplier, but if the supplier does not have enough goods inventory, the supplier needs to bear the risk of repurchase, if in the repurchase process. Among them, the residual value of the repurchased product is seriously inconsistent with the dealer's order quantity. To reduce its own losses, the supplier generally chooses to reject the credit risk considered by the repurchase bank, which means that when the supplier cannot provide the goods as agreed, the bank will obtain income through mortgage realization. Variable definition and description are shown in Table 2.

Here, we define the distribution function of the market demand *D* faced by dealers as the density function *F*(*x*), which satisfies the condition: *F* is single-increasing and differentiable and *F*(0) = 0, so that *F* = 1 − *F*(*x*), and then,

(1) $$\begin{array}{c} \mu =E\left(D\right)=\int_{0}^{+\propto }x\cdot f\left(x\right)\text{d}x,\\ S\left(Q\right)=\int_{0}^{Q}xf\left(x\right)\text{d}x+Q\int_{Q}^{+\propto }f\left(x\right)\text{d}x=Q-\int_{0}^{Q}F\left(x\right)\text{d}x. \end{array}$$

The prepayment financing business is a business established by the bank to grasp the information of each part of the supply chain and coordinate the relationship between the various parts. At the beginning of financing, the supplier and the distributor must sign a contract to ensure the supply of goods. In this process, if there are insufficient funds, you can use the advance account financing business to fight for investment from the bank. When the contract period is about to end, the dealer will repay the principal and interest of the financing to the bank; that is,

(2) $$\begin{array}{c} \frac{\text{d}S\left(Q\right)}{\text{d}Q}=1-F\left(Q\right)=\bar{F}\left(Q\right). \end{array}$$

When the market demand is insufficient, the repurchase amount is the remaining amount of the expected product at the end of the period.

(3) $$\begin{array}{c} y_{1}=y_{0}\left(1+r\right)=\left(uQ-C_{0}\right)\left(1+r\right). \end{array}$$

### 4.2. The Performance Difference between the Prepayment Financing Model and the Traditional Supply Chain Model

Under the prepayment financing model, the financing service provided by banks to dealers is based on the supplier's credit guarantee for repurchase. Therefore, this article focuses on the analysis of supply chain income considering the risk of default repurchase.

Assume that it is the critical point of market demand where the bank faces the risk of default repurchase; when the market demand *D* > *N* faced by the dealer, the bank can obtain the expected return, and when *D* < *N*, the supplier refuses to repurchase, and the bank will assume the supply losses caused by the breach of contract by the business. The expected income of the bank can be expressed as follows:

(4) $$\begin{array}{c} X\left(D\right)=E{\left(Q-D\right)}^{+}=Q-S\left(Q\right). \end{array}$$

After finishing, it is available as follows:

(5) $$\begin{array}{c} \Pi_{b}=\left\{\begin{array}{cc} y_{0}\cdot r+K-t, & D>N,\\ y_{0}\cdot r-\left(u-v\right)E{\left(Q-D\right)}^{+}+K-t, & D\leq N. \end{array}\right. \end{array}$$

Supplier's expected revenue sales revenue = sales cost − repurchase cost − repurchase revenue.

(6) $$\begin{array}{c} \Pi_{b}=\left(\left(uQ-C_{o}\right)\cdot r+K-t\right)\cdot P\left(D>N\right)\\ +\left[\left(uQ-C_{o}\right)\cdot r-\left(u-v\right)\cdot E{\left(Q-D\right)}^{+}+K-t\right]\cdot P\left(D\leq N\right)\\ =\left(uQ-C_{o}\right)\cdot r-\left(u-v\right)\int_{0}^{Q}F\left(x\right)\text{d}x\cdot P\left(D\leq N\right)+K-t. \end{array}$$

Available after finishing

(7) $$\begin{array}{c} \Pi_{N}=uQ-cQ-\left(u-v\right)E{\left(Q-D\right)}^{+}P\left(D>N\right)-0\cdot P\left(D\leq N\right). \end{array}$$

The dealer's expected revenue = sales revenue − sales cost − stock-out opportunity cost − loan interest and expenses.

(8) $$\begin{array}{c} \Pi_{H}=uQ-cQ-\left(u-v\right)E{\left(Q-D\right)}^{+}P\left(D>N\right)-0\cdot P\left(D\leq N\right)\\ =\left(u-c\right)Q-\left(u-v\right)\int_{0}^{Q}F\left(x\right)\text{d}x\cdot \left[1-P\left(D\leq N\right)\right]. \end{array}$$

Available after finishing

(9) $$\begin{array}{c} \Pi_{h}=p\cdot S\left(Q\right)-u\cdot S\left(Q\right)-g_{b}E{\left(D-Q\right)}^{+}-\left(uQ-C_{0}\right)\cdot r-K. \end{array}$$

Under the traditional supply chain, core suppliers rarely consider borrowing their own credit advantages to help dealers apply for financing services from banks. In this case, the supplier's expected revenue = sales revenue − sales cost.

(10) $$\begin{array}{c} \Pi_{h}=p\cdot S\left(Q\right)-u\cdot S\left(Q\right)-g_{k}E{\left(D-Q\right)}^{+}-\left(uQ-C_{0}\right)\cdot r-K\\ =\left(p-u+g_{h}\right)\left[Q-\int_{0}^{Q}F\left(x\right)\text{d}x\right]-g_{h}\cdot \mu -\left(uQ-C_{0}\right)\cdot r-K. \end{array}$$

The dealer's expected revenue type sales revenue = sales cost – stock-out opportunity cost.

(11) $$\begin{array}{c} \Pi_{h}=uQ^{*}-cQ^{*}=\left(u-c\right)Q^{*},\\ \Pi_{h}=pQ^{*}-uQ^{*}-g_{h}\left(D-Q^{*}\right)=\left(p-u\right)Q^{*}-g_{h}\left(D-Q^{*}\right). \end{array}$$

The bank did not receive interest income because it did not participate in the traditional supply chain service model, but in the process of business development, it will pay the cost *T* of information collection and credit evaluation of small and medium enterprises such as dealers.

In today's scarcity of resources, to improve resource utilization, high energy-consuming companies are looking for a transformation direction. The high-turnover, low-inventory marketing model is welcomed by many high-energy companies. This method can reduce the cost of storage for enterprises. In addition, waste of resources can be reduced. Some companies have adopted a variety of smart devices to strengthen the monitoring of each part of the industry chain to ensure real-time data, so that they can replenish resources and clean up inventory in a timely manner. For food production companies, the biggest problem they need to face during the production process is the storage of raw materials. Most food raw materials have a short shelf life. To ensure the absolute health of food materials, relevant departments also need to deal with food companies. The equipment and raw materials are monitored layer by layer. The monitoring process often takes a lot of time. During this time, the raw materials may be corrupted and deteriorated.

If Internet technology is applied to the processing and production process of food companies, it can directly improve the efficiency of production and operation without increasing costs. To study the growth of efficiency and revenue, this article will adopt the method of model construction (the following data are a simulation approximate variables).

(12) $$\begin{array}{c} \sum_{t=0}^{n}\frac{\text{NCP}t}{{\left(1+\text{IRR}\right)}^{t}}=0, \end{array}$$

where NCF is net cash flow of corporate purchase and sales collection, T is the time scale of the unit period, taking 15; and IRR is the internal rate of return (return) of the enterprise during the corresponding period.

The following article is based on the premise of not considering compound interest superposition (enterprise investment in reproduction) and compares the enterprise income before and after the enterprise achieves QC preproduction.

#### 4.2.1. The NCF Situation of the Company in the Three Sales Cycles under the Original Model

In the first production and operation model, under the original operating conditions, the ROCE before interest and tax before the company's inventory optimization is as follows:

(13) $$\begin{array}{c} \text{ROCE}=\frac{\text{IRR}\times 360}{15}=6\%\times 24=144\%. \end{array}$$

Under this production and operation model, if the company itself has sufficient funds, but the utilization rate is low, it will lead to an increase in costs and a decrease in revenue, which will harm the interests of the company.

If the company's funds are insufficient, to fill the gap of funds, the company often has the problem of inventory preparation. To solve this problem, it needs to continuously carry out financing activities in a short time. Assume that the short-term financing cost *R* is 10% (annualized), the financing and financial costs that a company needs to pay after completing 12 sales cycles in a year:

(14) $$\begin{array}{c} \text{Financing cost of funds occupied}=\frac{\left(N-1\right)\times \text{Quality inspection days}\times R}{360}. \end{array}$$

#### 4.2.2. NCF Situation of the Three Sales Cycles after the Company's Own Inventory Optimization

In the second production and operation model, the food company upgraded its own inventory management and used the method of purchasing raw materials in small batches and multiple batches, combined with its own production line capabilities, and carried out inventory optimization design. The achievable ROCE before interest and tax for a company is as follows:

(15) $$\begin{array}{c} \text{ROCE}=\frac{\text{IRR}\times 360}{15}=8\%\times 24=192\%. \end{array}$$

After inventory optimization, it can be simulated and calculated that the return on capital operation of the enterprise is 192%, which is an increase of 48% compared with the first operating model, but this is based on the optimization of capital utilization from the perspective of financial cost control. This is achieved by reducing the weighted operating costs (capital occupation) during the production cycle. Adopting this model is essentially a conservative management method based on financial concepts, and it cannot actually increase the growth of main business income, which fundamentally limits the production potential of the company; in addition, because the company fails to solve the problem of continuous production inventory preparation issues, companies still have short-term financing needs for operating liquidity.

#### 4.2.3. After Achieving QC, the NCF Situation of the Company's 3 Sales Cycles Are in the Third Production and Operation Mode

The food company entrusts the measurement and Testing Service Department of L company to be responsible for the quality inspection service of raw materials of its upstream purchasing unit before delivery. With the access to the enterprise port of the measurement and detection digital platform, the intelligent upgrading of the production equipment is completed by using the plug-in industrial control system (the cost of the control board is 600-1000 yuan). Since RFID is used to trace the raw materials of the tested batches in the delivery link, the traceability of the raw materials and product identities is realized. The raw materials are not required to be tested for the second time from the upstream delivery to the factory production link. Through the pre-QC, based on the traceability of product certification data, the problem of occupation of enterprise production inventory caused by “second inspection” is theoretically solved.  Figure 5 shows the situation of NCF after the optimization of the new production method in the industrial Internet of things environment and food companies.

The biggest difference between the third production mode and the first two production modes is that the increase in the rate of return on capital operations calculated under this mode is based on the premise that the company's own funds are sufficient and the production capacity can be improved. On the basis of no increase in operating costs, the actual revenue growth brought by the improvement of sales turnover efficiency has been realized.

From the comparison of the calculation results of the above models, it can be concluded that the pre-QC of raw materials realized through the intelligent transformation and upgrading of the equipment, on the one hand, under the optimized inventory management, reduces the financial cost of the enterprise and maximizes the capital utilization efficiency. The increase in corporate operating income is significantly increased. On the other hand, on the basis of matching the actual production capacity, the company's budget management can be further used to optimize order preparation to reduce the capital occupation caused by the production preparation. The changes in the specific income of the enterprise under the three production and sales conditions are compared, as shown in Table 3.

After the production line is intelligently upgraded, the intelligent remote control and monitoring realized by the enterprise greatly reduce the labor and management costs of the enterprise. From the perspective of management economics, because of the changes in production factors caused by the reduction in the marginal cost of unit production, enterprises can fully expand reproduction and further pursue profit maximization. Therefore, under this model, the actual profit growth of food companies based on their own development needs without increasing the company's operating costs (the cost of intelligent module transformation is lower) will far exceed 70%.

The core idea of supply chain finance is that this industrial chain involves the overall deployment of enterprises, to effectively use all funds in the enterprise and provide solutions for financing innovation through the flexible use of financial products, so that the industrial chain and related enterprises produce synergies and increase the competitiveness of the entire supply chain. Because it includes the entire process from raw materials to final products, it requires unified planning of logistics, capital flow, and information flow, so this provides a natural application scenario for the use of digital technology. As mentioned earlier in the service operation mechanism of using “Internet of Things technology” plus “Supply Chain Finance,” embedding industrial Internet of things technology in supply chain financial services can not only optimize risk management but also better obtain benefits. The upstream and downstream enterprises of the industrial chain perceive and provide the differentiated financial services required by the enterprises.

### 4.3. Analysis of Bank Financing Decisions in the Prepayment Financing Mode

The bank's decision to provide financial financing services must consider a variety of uncertain factors to determine whether to provide financing and loan services to the transaction partner, which reflects the balance between bank profits and credit risk. This section will establish a bank loan interest rate model with default risk based on the bank's expected profit analysis. In the form of passbook financing, it will study the main factors of supply chain finance that affect bank financing interest rates.

Suppose we consider bank financing services in the context of credit market competition. At this time, regarding the bank as a risk-seeking financial investor, there is no difference in identifying the investment risks of different projects. The financing services provided for them will meet the bank's expected return, which is equivalent to the average capital return in the capital market, which is

(16) $$\begin{array}{c} \Pi_{b}\left(r\right)=y_{0}\cdot r_{f}. \end{array}$$

Taking into account the supplier's risk of default, suppose that the contract expires and the supplier's order quantity is insufficient, which is lower than the quantity of the purchase contract, and the repurchase is refused, and the supplier defaults. Then, the bank has to bear the credit risk of supplier default and the loss of handling unsold goods; then,

(17) $$\begin{array}{c} \left(uQ-C_{0}\right)\cdot r-\left(u-v\right)\left[F\left(N\right)\cdot \left(Q-N\right)+\int_{0}^{N}F\left(x\right)\text{d}x\right]+K-t=\left(uQ-C_{0}\right)\cdot r_{f}. \end{array}$$

By organizing the above formula, you can get

(18) $$\begin{array}{c} r=r_{f}+\left(u-v\right)\frac{\left(1-\alpha \right)\cdot Q\cdot F\left(\alpha Q\right)+\int_{0}^{eQ}F\left(x\right)\text{d}x-K+t}{uQ-C_{0}},\;\alpha \in \left(0,1\right). \end{array}$$

The bank's financing interest rate has a huge impact on the development of banking business and the development of supply chain enterprises. The interest rate that the bank pays for the loan affects interest and credit risk, and the interest rate of the loan affects the financing cost of sellers, which in turn affects their net profit. To ensure that the loan interest rate is in line with the bank's own interests and that the creditor can pay the loan cost for the bank to any extent, the bank must adjust the borrowing cost.

Under the deposit financing model, the supplier promises to repurchase, but if the seller's order quantity is significantly lower than the agreed order quantity, the supplier will not repurchase. Therefore, in the bank's deposit financing model, the credit risk is mainly the supplier's repurchase default. The previously set loan form also reflects the supplier's repurchase rate, that is, reflects the corporate reputation. Here, we analyze the relationship between the two through the one-way loan of the loan interest rate to the corporate reputation.

(19) $$\begin{array}{c} \frac{\partial r}{\partial \alpha }=\frac{\left(u-v\right)}{uQ-C_{0}}+\left[Q\cdot \alpha \cdot \left(1-\alpha \right)f\left(\alpha Q\right)\right]>0. \end{array}$$

For banks, the rapid rise in credit rates means that suppliers are more likely to default. For suppliers' default risks, we can comprehensively evaluate factors such as their past transaction credit records and current product market demand conditions.

## 5. Analysis of the Research Results of the Supply Chain Financing Prepayment Model

### 5.1. Three-Party Cost-Benefit Analysis

When banks provide lenders with deposit funds, they should consider the supplier's repurchase risk. If the market demand of the enterprise is *X* > *N*, the bank will achieve the expected profit. On the contrary, when *X* < *N*, the supplier defaults and refuses to repurchase, and the bank bears the default loss for the unsold products. The expected return of the bank is as follows:

(20) $$\begin{array}{c} \Pi_{B}=\left[\left(uQ-C_{0}\right)\cdot r+K-t\right]\cdot P\left(D>N\right)+\left(\left(uQ-C_{0}\right)\cdot r-\left(u-v\right)\cdot E{\left(Q-D\right)}^{+}+K-t\right)\cdot P\left(D\geq N\right)\\ =2.5Q-0.25\int_{0}^{Q}F\left(x\right)\text{d}x-29. \end{array}$$

The supplier's expected benefits are as follows:

(21) $$\begin{array}{c} \Pi_{5}=uQ-cQ-\left(u-v\right)E{\left(Q-D\right)}^{+}P\left(D>N\right)-0\cdot P\left(D\leq N\right)=3Q-4.75\int_{0}^{Q}F\left(x\right)\text{d}x. \end{array}$$

The expected benefits of dealers are as follows:

(22) $$\begin{array}{c} \Pi_{G}=p\cdot S\left(Q\right)-u\cdot S\left(Q\right)-g_{b}E{\left(D-Q\right)}^{+}-\left(uQ-C_{0}\right)\cdot r-K=6.5Q-9\int_{0}^{Q}F\left(x\right)\text{d}x-95. \end{array}$$

Under the traditional supply model, banks are often afraid of small- and medium-sized enterprises in consideration of credit risk, so when they are unwilling to borrow, dealer *H* cannot get financing support from bank *M* and can only use his own funds to buy cars. The corresponding costs and benefits of the three parties are described as follows: supplier *T*'s expected benefits are as follows:

(23) $$\begin{array}{c} \Pi_{S1}=uQ^{*}-cQ^{*}=\left(u-c\right)Q^{*}=3Q^{*}. \end{array}$$

The expected benefits of dealer *H* are as follows:

(24) $$\begin{array}{c} \Pi_{G1}=pQ^{*}-uQ^{*}-g_{h}\left(D-Q^{*}\right)=\left(p-u\right)Q^{*}-g_{h}\left(D-Q^{*}\right)=9Q^{*}-120. \end{array}$$

Although banks do not belong to the traditional service supply chain and have no interest income, they still have to pay the cost *T* of information collection and credit review for SMEs, as shown as follows:

(25) $$\begin{array}{c} \Pi_{B1}=T=-8. \end{array}$$

The overall income of the supply chain under the deposit financing model is as follows:

(26) $$\begin{array}{c} \Pi_{1}=\Pi_{S}+\Pi_{G}+\Pi_{B}=120Q-14\int_{0}^{Q}F\left(x\right)\text{d}x-124,\\ \Pi_{2}=\Pi_{S1}+\Pi_{G1}+\Pi_{B1}=120Q^{*}-128. \end{array}$$

The maximum benefit of the overall supply chain is calculated as follows:

(27) $$\begin{array}{c} \text{Max}\left(\Pi_{2}\right)=12\times 12-128=16. \end{array}$$

In the case of deposit financing, banks provide financial support to dealers mainly because there is a funding gap in dealer purchases; that is, when the order quantity *D* < 15, dealers can purchase with their own funds without loan services.

(28) $$\begin{array}{c} \frac{\partial \Pi_{1}}{\partial Q}=12-14F\left(Q\right)>0. \end{array}$$

Through calculation,

(29) $$\begin{array}{c} \Pi_{1}=12\times 13-14\times 0.9175-124=19.155. \end{array}$$

### 5.2. Determination of Bank Loan Interest Rates

#### 5.2.1. Analysis of the Impact of Supplier Credit on Loan Interest Rates

The supplier's repurchase losses come from changes in market demand, so the actual quantity ordered by the distributor will be lower than the quantity stipulated in the contract. Assuming that the contract purchase quantity *D* between the supplier and the dealer is fixed, let *D* = 350; that is, under different market demand changes, the supplier will have different default probabilities.

(30) $$\begin{array}{c} r=r_{f}+\left(u-v\right)\frac{\left(1-\alpha \right)\cdot Q\cdot F\left(\alpha Q\right)+\int_{0}^{Q}F\left(x\right)\text{d}x-K+t}{uQ-C_{0}}. \end{array}$$

The model values are analyzed, and the calculation results are shown in Table 4.

#### 5.2.2. Analysis of the Impact of Financing Scale and Order Quantity on Bank Loan Interest Rates

As part of deposit financing, banks use the power and credit of core enterprises in the supply chain to reduce the credit rating and supervision costs of small- and medium-sized enterprises. The larger the dealer's financing scale, the more profit the bank can make.

(31) $$\begin{array}{c} F\left(x\right)=\int_{-\infty }^{\infty }\frac{1}{\sqrt{2\pi \sigma }}e^{-{\left(x-\mu \right)}^{2}/2\sigma^{2}}. \end{array}$$

In the same way, *D* can calculate the demand between different markets, which can get D's business scope, as shown in Table 5.

In the interval (35–60), the probability will also reach 70%. On this basis, the interval value of the dealer's purchase quantity is found, and a rough division of other small probability events is made. The interval division of order quantity is shown in Table 6.

The loan interest rate issued by dealers in different loan ranges is *R*. On the premise of not exceeding the upper limit of the loan range, the loan interest rate of the upper limit of the loan range is used as the calculation basis, as shown in Table 7.

#### 5.2.3. Comparative Analysis of Costs and Benefits under the Two Supply Chain Models

(1) Comparative analysis of the overall cost and benefit of the supply chain under the two modes
Under the supply chain model, tripartite revenue = bank revenue + supplier revenue + distributor revenue.
  (32) $$\begin{array}{c} \Pi_{1}=\Pi_{b}+\Pi_{H}+\Pi_{h}\\ =\left(p+g_{h}-u\right)\cdot S\left(Q\right)-\left(u+c\right)Q-\left(u-v\right)\left[Q-S\left(Q\right)\right]-g_{h}\mu -t\\ =\left(p+g_{h}-c\right)\cdot Q-\left(p+g_{h}-v\right)\int_{0}^{Q}F\left(x\right)\text{d}x-g_{h}\cdot \mu -t. \end{array}$$
Traditional supply chain tripartite revenue = supplier revenue + distributor revenue − bank costs.
  (33) $$\begin{array}{c} \Pi_{2}=\Pi_{H}+\Pi_{h}-T=\left(p+g_{h}-c\right)\cdot Q-g_{h}\cdot D-T=\left(p+g_{h}-c\right)\cdot Q-g_{h}\cdot D-T. \end{array}$$
(2) Comparative analysis of tripartite cost and benefit of supply chain under two modes
  (a) The differences in bank income between the two models are as follows:
    (34) $$\begin{array}{c} \Delta \Pi_{b}=\left(uQ-C_{0}\right)\cdot r-\left(u-v\right)\int_{0}^{Q}F\left(x\right)\text{d}x\cdot P\left(D\leq N\right)+K-\left(t-T\right). \end{array}$$
  The difference in bank income mainly comes from the interest generated by loans, income from financing recovery expenses, and the cost of credit valuation.
  (b) The difference in supplier income between the two models is as follows:
    (35) $$\begin{array}{c} \Delta \Pi_{H}=\left(u-c\right)\cdot \left(Q-Q\right)-\left(u-v\right)\int_{0}^{Q}F\left(x\right)\text{d}x\cdot \left[1-P\left(D\leq N\right)\right]. \end{array}$$
  The difference in supplier income is mainly due to the fact that dealers can take loans first and then purchase goods. When the number of products sold increases, their income will increase. At the same time, the risk of repurchase can be controlled within a certain range to cause greater changes in income.
  (c) The difference in dealer income between the two models is as follows:
    (36) $$\begin{array}{c} \Delta \Pi_{b}=\left(\left(p-u\right)\left(Q-Q\right)+g_{h}\left(Q+Q\right)-2\;D\right)-\left(uQ-C_{0}\right)\cdot r-\left(p-u+g_{b}\right)\int_{0}^{Q}F\left(x\right)\text{d}x-K. \end{array}$$
  The income difference of distributors is mainly due to the reduction in bank loan interest rates and sufficient funds. They can purchase products in large quantities, thereby obtaining preferential prices and reducing purchase costs.

## 6. Conclusion

With the liberalization of national policies, the rapid progress of information technology and the increasing improvement of communication infrastructure have broken the previous limitation that only traditional financial institutions were able to become the main body of supply chain financial products and services. In the supply chain, the core enterprises with strong control and information processing capabilities develop the provision of financial services and provide a good environment for innovation and development. At the moment when we are advocating “mass entrepreneurship and innovation,” we should always stay awake about some of the current phenomena. Because of the huge demand for the supply chain finance market in emerging industries, big data analysis plus supply chain finance has attracted increasing attention as a new capital flow model. The market will be popular afterwards. Given the weak growth of traditional enterprises, supply chain financing has gradually become a new business growth center. In recent years, these supply chains have the most potential for development in the field of bank transaction financing innovation. The supply chain financing included in the supply chain relies on the reputation of core enterprises to provide credit support for small and medium enterprises upstream and downstream of the supply chain to solve the problem of financing difficulties for small- and medium-sized enterprises, which not only promotes core enterprises and related upstream and downstream enterprises. Long-term strategic collaboration has also improved the overall competitiveness of the supply chain.

## Figures and Tables

**Figure 1:** Accounts receivable pledge process.

**Figure 2:** Confirmed warehouse financing process.

**Figure 3:** Mapping relationship among supply chain performance indicators, factors, and problems.

**Figure 4:** Technical route of intelligent analysis method of supply chain performance.

**Figure 5:** NCF situation of the company's 3 sales cycles after the original and the company's own inventory optimization and after the realization of QC (quality control).

**Table 1:** Advantages of data acquisition in the production environment of industrial Internet of things.

No.	Industrial basic service module	Principles of risk control optimization
1	Production process monitoring	These data directly reflect the company's production process, production process, and production safety status and are the most true underlying data of the company
2	Online product testing	Through the online testing data of the product, according to the technical indicators of the product, the technical level of the company in the segmented industry is obtained, and then, the competitiveness of the industry in which the company is located can be judged
3	Informationized inventory management	The inventory data of raw materials and finished products of enterprises can be used for supporting analysis on the financial statement data provided by the enterprises based on the calculated turnover rate of the focus enterprise's inventory and order scale status

**Table 2:** Variable definition and description.

Variable definitions	Variable description
*y *_1_	Bank's ending income
*C *_0_	Dealer's own funds
*r*	Bank loan interest rate
*U*	Supplier sales price
*C*	Supplier production cost
*V*	Unit residual value of products purchased by suppliers (*v* ≦ *u*)
*P*	Dealer sales price
*Q*	Dealer order quantity
*D*	Market demand faced by dealers
*g*_*k*_	The unit penalty cost of goodwill caused by the dealer's shortage
*K*	Fee income from services provided by banks (fixed value)
*T*	The sum of other related costs and risks borne by banks under the traditional supply chain
*t*	The sum of other related costs and risks borne by banks under supply chain finance (*t* < *T*)

**Table 3:** Comparison of corporate earnings under three inventory management models.

No.	Production and business model	ROCE (%)	Main business income growth rate
1	Original production status	144.0	**—**
2	Enterprise's own inventory management optimization	192.0	**—**
3	After realizing QC front	240.0	65.7%

**Table 4:** Impact of corporate credit on bank loan interest rates.

*r*	0–0.05	0.05–0.10	0.1–0.15	0.15–0.20
*μ*	0.1055	0.1068	0.1085	0.1104

**Table 5:** Interval division of market demand *D*.

D probability of occurrence	100%	90%	80%	70%	60%	50%	40%	30%	20%	10%
	0–80	0–50	0–43	0–38	0–34	0–30	0–26	0–22	0–17	0–12

**Table 6:** Interval division of order quantity *Q*.

*D* order probability	0.1	0.4	0.4	0.1
	(0, 12]	(12, 30]	(30, 50]	(50, 80]

**Table 7:** Examples of loan interest rates.

	(0, 450]	(450, 950]	(950, 1700]
(0, 12]	No loan required	No loan required	No loan required
(12, 30]	0.1055	No loan required	No loan required
(30, 50]	0.1106	0.1050	No loan required
(50, 80]	0.1212	0.1100	0.1056

## Data Availability

The data used to support the findings of this study are available from the corresponding author upon request.
